# On the Use of Wavelet Domain and Machine Learning for the Analysis of Epileptic Seizure Detection from EEG Signals

**DOI:** 10.1155/2022/8928021

**Published:** 2022-02-25

**Authors:** K. V. N. Kavitha, Sharmila Ashok, Agbotiname Lucky Imoize, Stephen Ojo, K. Senthamil Selvan, Tariq Ahamed Ahanger, Musah Alhassan

**Affiliations:** ^1^Department of Communication Engineering, School of Electronics Engineering, Vellore Institute of Technology, Vellore, Tamil Nadu, India; ^2^Department of Control and Automation, School of Electrical Engineering, Vellore Institute of Technology, Vellore, Tamil Nadu, India; ^3^Department of Electrical and Electronics Engineering, Faculty of Engineering, University of Lagos, Akoka, Lagos 100213, Nigeria; ^4^Department of Electrical Engineering and Information Technology, Institute of Digital Communication Ruhr University, 44801 Bochum, Germany; ^5^Department of Electrical and Computer Engineering, College of Engineering, Anderson University, Anderson, SC, USA; ^6^Prince Shri Venkateshwara Padmavathy Engineering College, Chennai, Tamil Nadu, India; ^7^College of Computer Engineering and Sciences, Prince Sattam Bin Abdulaziz University, Al-Kharj, Saudi Arabia; ^8^Electrical Engineering Department, School of Engineering, University of Development Studies, Nyankpala Campus, Nyankpala, Ghana

## Abstract

Epileptic patients suffer from an epileptic brain seizure caused by the temporary and unpredicted electrical interruption. Conventionally, the electroencephalogram (EEG) signals are manually studied by medical practitioners as it records the electrical activities from the brain. This technique consumes a lot of time, and the outputs are unreliable. In a bid to address this problem, a new structure for detecting an epileptic seizure is proposed in this study. The EEG signals obtained from the University of Bonn, Germany, and real-time medical records from the Senthil Multispecialty Hospital, India, were used. These signals were disintegrated into six frequency subbands that employed discrete wavelet transform (DWT) and extracted twelve statistical functions. In particular, seven best features were identified and further fed into k-Nearest Neighbor (kNN), naïve Bayes, Support Vector Machine (SVM), and Decision Tree classifiers for two-type and three-type classifications. Six statistical parameters were employed to measure the performance of these classifications. It has been found that different combinations of features and classifiers produce different results. Overall, the study is a first attempt to find the best combination feature set and classifier for 16 different 2-class and 3-class classification challenges of the Bonn and Senthil real-time clinical dataset.

## 1. Introduction

Epilepsy is a brain disorder that includes repeated seizures in the brain due to uncontrolled electrical movement. It results in uninhibited jerking movement and momentary loss of consciousness. It is potentially life-threatening as it causes malfunction of the brain and lung, heart failure, and unexpected deaths caused by accident. Therefore, it is imperative to diagnose epilepsy [1]. The signal that records electrical movement and activity in the brain is the electroencephalogram (EEG) signal. Electrodes are placed on various parts of the scalp during this procedure and produce multichannel data. Since it is a noninvasive and inexpensive method, it serves as a vital data resource in neurological diagnosis such as seizure detection [1, 2]. Typically, medical personnel collect recordings by visually inspecting the long-term EEG. This method consumes time, is cumbersome and prone to errors, and requires a certain level of human expertise. Thus, an automated epilepsy seizure detection framework is needed.

This tedious nature of reading EEG recordings by doctors to determine epileptic conditions has necessitated research into more straightforward, quicker, and more efficient methods of detecting epileptic conditions. In [3], a pattern recognition study was conducted using time-domain (TD) functions for detecting epileptic seizures, which includes waveform length (WL), some slope sign changes (SSC), and many zero-crossings (ZC) that are derivative of filtered EEG data and discrete wavelet transform (DWT) of filtered EEG data for the detection of epileptic seizures. Therefore, the performance of time-domain features was studied based on the support vector machines (SVM) classifiers and naïve Bayes (NB). With direct and DWT-based TD functions, the results revealed that the suggested technique should reach the best accuracy of 100 percent for regular eyes open and epileptic datasets.

In [4], it is imperative to use the combination of electroencephalogram (EEG) with the technique of deep learning computation to diagnose epileptic seizures, as highlighted in the study. This study emphasized designing and evaluating seizure detection using the deep convolution neural network-based classifier. The outcome proposed was to determine the most accurate seizure detection, and it was classified into three methods. 99.21% was the highest average classification accuracy, which was proposed to be the FT-VGG16 classifier using the accuracy data with previous studies of the same set of data. The outcome shows that comparing the signal-to-image conversion method and accuracy data model surpassed all earlier investigations in the vast majority. Furthermore, to discover the most improved classification accuracy and the EEG frequencies feature, the SHapley Additive exPlanations (SHAP) analysis approach was used.

In [5], the Bonn dataset was used to evaluate the new suggested technique for automatically recording epileptic electroencephalograms. This is based on approximated entropy and repetitive mixed quantification analysis, leveraging a convolution neural network. The results revealed that approximation entropy and recurrence quantification effectively detect epileptic seizures. 92.17%, 91.75%, and 92.00% show the recurrence rate of attainment of sensitivity and accuracy, respectively. The classic recordings automatically differentiate seizure electroencephalogram from convolutional neural networks, especially when combined with the approximate entropy and recurrence quantification analysis features. The results reached 98.84%, 99.35%, and 99.26%. Several other works in this domain all point to the fact that automatic detection of epileptic conditions can be a possibility, thus ruling out the tedious task of doctors inspecting EEGs. These tools would be helpful in epilepsy clinical diagnosis and therapy.

In providing an accurate solution to the problem of an epileptic seizure, several algorithms have been proposed, and they provide several levels of accuracy. In [6–8], several time-frequency domain algorithms were introduced for the accurate characterization of epileptic seizures from collected EEG signals. Two of the algorithms are short-time Fourier transform and multiwavelet transform. The two algorithms provided satisfactory results upon validation. Discrete wavelet transform was employed in [9] for epileptic seizure detection. This method was primarily used to extract features from the EEG signals and carry out the principal component analysis, independent component analysis, and, lastly, the linear discriminant analysis, which was introduced to reduce the dimensions of the various signals and for straightforward representation. Support vector regression machine learning-based model was then employed to classify the mixed EEG signals in the multidimensional plane.

As introduced, the Support Vector Machine is efficient for signal classification, but that does not come without the challenges of selecting the optimal number of parameters. Setting the proper parameter is crucial to achieving high accuracy in detecting epileptic seizures. This hyperparameter tuning and selection makes particle swarm optimization and genetic algorithms highly accurate. The detection of epileptic seizures must be done accurately and efficiently, and this is why machine learning algorithms have been recently introduced. The large volume of the dataset used in EEG signals can be processed accurately with the algorithms.

Also, the robust network architecture that ML algorithms provide makes them scalable and useful when characterizing EEG signals. The epileptic seizure detection must be performed with the lowest false negative and false positive. ML algorithms have been introduced to ensure this efficiency and accuracy in feature characterization. The digital wavelet transformation (DWT) introduced in [9, 10] was able to handle the problem of spikes in epileptic seizures. The DWT algorithm can handle the spikes through the localization of these transient occurrences. The algorithm prevents the generalization of the spike occurrences and thus reduces or minimizes any form of error at that particular time during the signal characterization process.

The detection of epileptic seizures was introduced using hybrid methods [11]. The generic algorithm was embedded into fuzzy logic and characterized both epileptic and nonepileptic signals. Various risk assessments to both the two signal characterizations (epileptic and nonepileptic) were provided by fusing the data into the genetic algorithm to make accurate predictions. Another hybrid method was introduced in [12], in which computational intelligence was integrated with a genetic algorithm to ensure optimal characterization of EEG signals. The entire dataset was divided into training and validation datasets. Features were extracted from the datasets and used to train the genetic algorithm. The validation datasets were then used to validate the trained model. The genetic algorithm-based model was able to detect epileptic seizures accurately. Hybrid models work efficiently and can adequately compensate for the deficiencies in each base model to produce a single model with high accuracy. For this particular base model, the accuracy largely depends on the proper tuning of the parameters of the genetic algorithm.

In [13], another model stationary wavelet transform was introduced and employed to detect an epileptic seizure. This presented algorithm properly captured points on the edge of the signal which are stationary at all points. The ability to capture these stationary points reduces the probability of error. This is because the points on the wavelet that would have been normally left unaccounted for have now been adequately represented with the aid of this stationary wavelet algorithm. It was applied to both epileptic and nonepileptic signals under varying conditions to determine its optimization level. The stationary wavelet algorithm is also efficient for handling the data points along rough edges that could negatively affect the seizure detection algorithm. The stationary points for the nonepileptic signals present some form of complexities. Still, they could also be handled appropriately with the stationary wavelet transformation for linear signals and nonlinear signals.

An algorithm was given to detect epileptic seizures in [14]. The study used data from both epileptic patients and those who are not epileptic patients to develop the framework. The authors then classified the sample features into various datasets using linear and nonlinear classifiers. The linear classifier handled the measurements taken from nonepileptic patients, while the nonlinear classifiers were used to classify epileptic patients. Digital wavelet transformation was then later used to analyze seizure detection. The datasets were also divided into the training and the test datasets to ensure proper characterization in all cases. While the detection algorithm was developed with the training dataset, the testing was carried out with the test datasets to prevent overfitting and reduce the number of outliers. Several other algorithms have been developed and used in epileptic seizure detection, but some present one form of limitation or the other. The concern is not just in the development of an algorithm. The focus should be on optimization and accurate characterization so that seizure detection can be done with the lowest possible form of error.

This work combines the wavelet domain and machine learning approach to identify epileptic seizures. Time-frequency analysis is carried out on EEG signals as they are nonlinear, nonstationary, and complex. There are many methods for performing time-frequency analysis. In this study, the discrete wavelet transform technique is adopted. Extracting the hidden characteristics of the signal is done by using feature extraction, which helps in inspecting the signal. These derived features are fed into classifiers that differentiate between healthy and seizure signals. The classifiers used are k-Nearest Neighbor (kNN), Support Vector Machine (SVM), naïve Bayes, and Decision Tree classifier [15, 16]. The performance of these classifiers is measured using statistical parameters.

The remainder of this work is structured as follows.  Section 2 presents the methodology. The results and discussions are given in Section 3. The comparison with other existing state-of-the-art developments is given in Section 4, and the conclusion is given in Section 5.

## 2. Methods

The EEG data is fragmented into six frequency subbands using the discrete wavelet transform. The essential characteristics, such as mean average power, lowest coefficient, average value, and highest coefficient, are removed and inputted into naïve Bayes, SVM, Decision Tree classifiers, and kNN. The computation performance is done for each classifier and feature. The proposed framework is indicated in Figure 1.

### 2.1. Bonn University Dataset

This data is available on the website of the Department of Epileptology, Bonn University, Germany [15]. This is a single-channel data provided solely for research purposes. The record contains five datasets named as set A to set E. Each set of data has 100 samples. The time taken is 23.6 s for 100 EEG segments recorded on the head's surface via a single channel. Five healthy volunteers were chosen for clusters A and B, and the EEG signals were recorded with keen observation, respectively. For cluster C, there are the patients who do not have the epileptic attack at hemisphere hippocampal formation, and, for cluster *D*, the epileptogenic zone is where the recording took place. Set E of the EEG signal was recorded, while the patients were experiencing an epileptic attack. A 12-bit A/D converter with a 173.61 Hz sampling frequency is used for digitizing the data. Therefore, each EEG segment is found to contain 4096 points of sampling. The graphs of EEG signals are plotted and presented in Figure 2.

### 2.2. Real-Time Clinical Dataset

Real-time multichannel clinical data were acquired from six healthy patients and six epileptic patients from Senthil Multispecialty Hospital in Erode, Tamil Nadu, India. The data was 21-channel EEG data. The epileptic signal was recorded during the preseizure period. The sampling frequency is maintained at 256 Hz.

### 2.3. Preprocessing of Signal Using DWT

The Fast Fourier Transform (FFT) for frequency-domain analysis is applied in many applications. But, for biomedical signals such as EEG, the usage of FFT is restricted, since they include uneven patterns and are also nonstationary. The only time-domain analysis will not yield information regarding the frequency of the pattern. Therefore, the time-frequency analysis is applied for preprocessing the signal. Discrete wavelet transform is a widely used time-frequency analyzer for biomedical signals as it prefers variable window sizes. The DWT algorithm uses low-pass (LP) and high-pass (HP) quadrature mirror filters.

The input signal is routed through the low- and high-pass filters to produce the approximate (A1) coefficient and their outputs detailed (D1) coefficient. The result obtained from the high-pass filter is provided to another filter of quadrature mirror type, and the process is repeated to determine the coefficients of the subsequent level. Every decomposition process leads to doubling the frequency resolution because of filtering and halved through downsampling.

This work uses Daubechies order-4 wavelet function due to its orthogonal features and filtering efficiency. The necessary statistical features are acquired from the subbands frequency.

### 2.4. Statistical Features from Discrete Wavelet Transform (DWT) Coefficients

The following features were extracted.

*Mean Average Value* (*MAV*). MAV relates to the information frequency of the signal and can be determined from the following equation:

(1) $$\begin{array}{c} \text{MAV}=\frac{1}{N}\sum_{i=1}^{N}\left|x_{i}\right|. \end{array}$$

*Maximum Coefficient*. The maximum coefficient measures the maximum frequency value for a given sample.

*Minimum Coefficient*. The minimum coefficient measures the minimum value of frequency for a given sample.

*Standard Deviation* (*STD*). Standard deviation relates to the proportionate changes in the frequency signal and is given by the following equation:

(2) $$\begin{array}{c} \text{SD}=\frac{1}{N-1}\sum_{i=1}^{N}\left(x_{i}-\mu \right).^{2} \end{array}$$

*Average Power*. Average power represents information about the frequency content of the signal and is determined by the following equation:

(3) $$\begin{array}{c} \text{AVP}=\frac{1}{N}\sum_{i=1}^{N}\left|x_{i}\right|.^{2} \end{array}$$

*Shannon Entropy*. The expression of Shannon entropy offers an easy mode to determine the average number of bits necessary to encode a string of symbols. It is given by the following equation:

(4) $$\begin{array}{c} H\left(X\right)=-\sum_{i=0}^{N-1}p_{i}\log_{2}p_{i}. \end{array}$$

*Approximate Entropy* (*ApEn*). The extent of regularity and unpredictability of fluctuations over time-series data can be quantified by approximate entropy, ApEn (*m*, *r*, *N*). The parameters *m* and *r* are the run length and tolerance window input parameters, respectively. The parameter *N* is the number of points of the time series.

### 2.5. K-Fold Cross-Validation

10-fold cross-validation is used in this study to get reliable results. The original sample is divided into 10 subsamples. The 9 subsamples are used as training datasets, and one subsample is used as testing dataset. It is then repeated 10 times. In this way, each dataset is trained 9 times and tested one time. The 10 results obtained are then averaged to give a single estimated accuracy. This validation is applied to SVM, KNN, naïve Bayes, and Decision Tree classifier.

### 2.6. Support Vector Machine (SVM) Classifier

SVM is a binary classifier model based on a machine learning algorithm. In this format, a training dataset is classified into two groups so that the division is as wide as possible. The machine learning [46] algorithm generates a plot of hyperplane, which distributes the two groups using the training dataset. From the plot, a set of data is considered nonsensitive if the hyperplane is closer to that data. Thus optimal hyperplane is chosen, which is farthest from the data points. The optimal hyperplane is used to classify the testing dataset.

The equation of hyperplane is

(5) $$\begin{array}{c} f\left(x\right)=\beta_{0}+\beta^{T}x, \end{array}$$

where *β* is the weight vector and *β*_0_ is the bias vector. An infinite number of hyperplanes can be obtained by varying the two parameters. The condition for optimal hyperplane is

(6) $$\begin{array}{c} \;\beta_{0}+\beta^{T}x=1, \end{array}$$

where *x* represents the support vector, the training set closest to the hyperplane.

### 2.7. k-Nearest Neighbor (kNN) Classifier

kNN is a nonparametric and nonlinear classifier. It is used for relatively larger training sets. The similarities between the training and testing [47] sets are considered for the measure. The class having the majority in the nearby “k” datasets is assigned to the test/unknown dataset. The dataset “nearness” is measured using Euclidean distance given by

(7) $$\begin{array}{c} \text{ED}=\;\sqrt{{\sum_{i=1}^{n}\left(Y_{1i}-Y_{2i}\right)}^{2}}, \end{array}$$

where *Y*_1*i*_=(*y*_11_, *y*_12_,…, *y*_1*n*_) and *Y*_2*i*_=(*y*_21_, *y*_22_,…, *y*_2*n*_).

The value of *k* should be a positive integer. In this study, the value of *k* is 3.

### 2.8. Naïve Bayes (NB) Classifier

This classifier is based on Bayesian theory and is a probabilistic classifier. It is also based on the assumption that each class feature is independent of any other feature. The NB classifier needs less training data.

Assuming *D* as a training set for *n* number of classes and *Y* as the attribute vector and associated class labels, the class with the highest posterior probability to which attribute *Y* belongs to is given by

(8) $$\begin{array}{c} P\left(C_{i}|Y\right)>P\left(C_{j}|Y\right)\text{ for}1\leq j\leq n,\;j\neq i, \end{array}$$

where

(9) $$\begin{array}{c} P\left(C_{i}|Y\right)=\;\frac{P\left(Y|C_{i}\right)\;P\left(C_{i}\right)}{P\left(Y\right)}\;, \end{array}$$

by Bayes theorem.

Here *P*(*C*_*i*_) represents the class probabilities, *P*(*Y*) is the prior probability of Y, *P*(*C*_*i*_*|Y*) is the posterior probability, and *P*(*Y|C*_*i*_) is the posterior probability of *Y* conditioned on *C*_*i*_.

### 2.9. Decision Tree (DT) Classifier

DT is a predictive modelling approach widely used in data mining, statistics, and machine learning algorithms. Tree models are used where the target variable is assigned with continuous values. The Decision Tree leaves represent the class labels, and the branches represent a combination of features that lead to those class labels.

### 2.10. Statistical Parameter

The performances of the four classifiers are evaluated using six parameters, namely, accuracy, specificity, sensitivity, positive predicted value (PPV), negative predicted value (NPV), and Mathews correlation coefficient (MCC) [4, 5]. These parameters are mathematically defined as follows:

Accuracy:

(10) $$\begin{array}{c} \mathrm{accuracy}\left(\%\right)=\frac{\mathrm{CCP}}{\mathrm{TPT}}\mathrm{\times 100\%}. \end{array}$$

Sensitivity:

(11) $$\begin{array}{c} \mathrm{sensitivty}\left(\%\right)=\frac{\mathrm{TP}}{\mathrm{TP+FN}}\mathrm{\times 100\%}. \end{array}$$

Specificity:

(12) $$\begin{array}{c} \mathrm{specificity}\left(\%\right)=\frac{\mathrm{TN}}{\mathrm{TN+FP}}\mathrm{\times 100\%}. \end{array}$$

Positive predictive value (PPV):

(13) $$\begin{array}{c} \mathrm{PPV}\left(\%\right)=\frac{\mathrm{TP}}{\mathrm{TP+FP}}\mathrm{\times 100\%}. \end{array}$$

Negative predictive value (NPV):

(14) $$\begin{array}{c} \mathrm{NPV}\left(\%\right)=\frac{\mathrm{TN}}{\mathrm{TN+FN}}\mathrm{\times 100\%}. \end{array}$$

Mathews correlation coefficient (MCC):

(15) $$\begin{array}{c} \mathrm{MCC}=\frac{\mathrm{TP\times TN}-\mathrm{FP\times FN}}{\sqrt{\left(\mathrm{TP}+\mathrm{FP}\right)\left(\mathrm{TP}+\mathrm{FN}\right)\left(\mathrm{TN}+\mathrm{FP}\right)\left(\mathrm{TN}+\mathrm{FN}\right)}}, \end{array}$$

where CCP denotes correct classified patterns, and total patterns are denoted as TPT. TP denotes true positive, FN denotes false negative, FP denotes false positive, and TN denotes a true negative.

## 3. Results and Discussions

### 3.1. Results from the University of Bonn Dataset

The datasets from sets A, B, C, D, and E are decomposed into different subbands. The different frequency subbands are D1 (43.4–86.8 Hz), D2 (21.7–43.4 Hz), D3 (10.85–21.7 Hz), D4 (5.42–10.85 Hz), D5 (2.70–5.43 Hz), and A5 (0–2.70 Hz). Since the most useful information is available in subbands D3–D5 and A5, only they are considered [10]. Features such as Mean Absolute Value, maximum coefficients, minimum coefficients, Standard Deviation, average power, Shannon entropy, and approximate entropy are derived from subbands D3, D4, D5, and A5 for five datasets A, B, C, D, and E.

Sixteen cases are considered, including 2 class classifications and 3 class classifications on data readily available from the University of Bonn, Germany. 7 features were obtained in the study. However, the number of features generated for each EEG signal should be 4 x 7 = 28. For every 100 signals of datasets A to E, 28 features were generated. In each case, 10-fold cross-validation is applied, dividing whole data into 10 equal parts, where 9 data parts are used for training against 1 used for testing purposes. The SVM, KNN, naïve Bayes, and Decision Tree classifiers are then fed the following training and testing sets, and performance measures such as Accuracy, Specificity, Sensitivity, Positive Predicted Value, Negative Predicted Value, and Mathews Correlation coefficients are obtained.

From Table 1, we can observe the result for 16 different classifications for the SVM classifier. For A-E classification, estimated entropy from the D5 frequency subband provides the highest level of accuracy of 100%. Similarly, for B-E classification, minimum coefficients extracted from D3, D4, and A5 frequency subbands give only 90%, 91%, and 92% accuracy, respectively, but approximate entropy extracted from D5 frequency subband gives the highest accuracy of 99.5%. For C-E classification, in D4 frequency subband, maximum coefficient gives the highest accuracy of 98%. For D-E classification, in the D3 frequency subband, MAV gives the best accuracy of 96%. For AB-E classification, in the D5 frequency subband, approximate entropy provides the highest level of accuracy of 99.67%. For AC-E classification, in the D5 frequency subband, MAV provides the highest level of accuracy of 98.66%. For AD-E classification, in the D3 frequency subband, MAV provides the highest level of accuracy of 98%. For BC-E classification, in the D3 frequency subband, the minimum coefficient gives an accuracy of 92.6%. For BD-E classification, in the D5 frequency subband, MAV provides the highest level of accuracy of 96.3%. For CD-E classification, in the D3 frequency subband, MAV gives the highest accuracy of 98%. For ABC-E classification, in the D5 frequency subband, MAV gives the highest accuracy of 99%. For ABD-E classification, in the D5 frequency subband, MAV gives the highest accuracy of 97%. For ACD-E classification, in the D3 frequency subband, MAV gives the highest accuracy of 98.25%. For BCD-E, in the D5 frequency subband, MAV gives the highest accuracy of 97%. For ABCD-E classification, in the D3 frequency subband, the minimum coefficient gives the best accuracy of 100%. For AB-CD classification, in the D3 frequency subband, approximate entropy gives an accuracy of 80%. Moreover, we can infer that the feature that provides SVM the best result is the Mean Absolute Value. The highest accuracy is achieved for A-E and ABCD-E classification, which is 100%. The lowest classification accuracy is achieved for AB-CD classification.

From Table 2, we can observe the result for 17 different classifications for the kNN classifier. For A-E classification, approximate entropy from the D5 frequency subband gives the highest accuracy of 100%. For B-E classification, maximum and minimum coefficients extracted from D3, D4, and A5 frequency subbands give poor results, but MAV extracted from D5 gives the best result of 100%. For C-E classification, in the D3, D4, and D5 frequency subbands, STD gives the highest accuracy of 98%, and in the A5 frequency subband, ApEp gives the accuracy of 79.5%. For D-E classification, in the D3 frequency subband, MAV gives the best accuracy of 97%. For AB-E classification, in the D5 frequency subband, MAV gives the highest accuracy of 100%. For AC-E classification, in the D3 frequency subband, STD gives the highest accuracy of 98.7%. For AD-E classification, in the D3 frequency subband, MAV gives the highest accuracy of 98%. For BC-E classification, in the D5 frequency subband, MAV gives a better result. The highest accuracy achieved for A-E, B-E, AB-E, and ABCD-E classification is 100%. The lowest classification accuracy is achieved for AB-CD and AB-CD-E classification, with the highest accuracy of 98.6%. For BD-E classification, in the D5 frequency subband, Shannon entropy gives the highest accuracy of 95.33%. For CD-E classification, in the D3 frequency subband, MAV gives the highest accuracy of 97.66%. For ABC-E classification, in the D5 frequency subband, MAV gives the highest accuracy of 99%. For ABD-E classification, in the D5 frequency subband, MAV provides the highest level of accuracy of 96.5%. For ACD-E classification, in the D3 frequency subband, Shannon entropy provides the highest level of accuracy of 98%. For BCD-E classification, in the D5 frequency subband, MAV provides the highest level of accuracy of 97%. For ABCD-E classification, in the D3 frequency subband, the minimum coefficient gives the best accuracy of 100%. For AB-CD classification, in the D5 frequency subband, MAV gives the best accuracy of 75%. For AB-CD-E classification, in the D5 frequency subband, Shannon entropy gives the best accuracy of 75%. Moreover, we can infer that Mean Absolute Value and Shannon entropy are the features that offer the best result for kNN.

From Table 3, we can observe the results for 16 different classifications for the naïve Bayes classifier. For A-E classification, MAV from the D5 frequency subband gives the highest accuracy of 100%. For B-E classification, the minimum coefficient extracted from D3, average power extracted from D4, and ApEp extracted from A5 frequency subband give poor results. Still, MAV extracted from D5 gives the best result of 99.5%. For C-E classification, in D3, D4, D5, and A5 frequency subbands, the STD has been extracted, and the highest accuracy of 100% has been attained only in the D5 frequency subband. For D-E classification, in the D3 frequency subband, MAV gives the best accuracy of 97.5%. For AB-E classification, in the D5 frequency subband, STD provides the highest level of accuracy of 99.7%. For AC-E classification, in the D3 frequency subband, STD provides the highest level of accuracy of 98.7%. For AD-E classification, in the D3 frequency subband, MAV provides the highest level of accuracy of 98%. For BC-E classification, in the D5 frequency subband, ApEp provides the highest level of accuracy of 98.7%. For BD-E classification, in the D5 frequency subband, ApEp gives the maximum accuracy of 96%. For CD-E classification, in the D3 and D4 frequency subbands, MAV gives the maximum accuracy of 97.7%. For ABC-E classification, in the D5 frequency subband, MAV gives the maximum accuracy of 99%. For ABD-E classification, in the D5 frequency subband, ApEp gives the maximum accuracy of 96.25%. For ACD-E classification, in the D5 frequency subband, ApEp gives the maximum accuracy of 97.6%. For ABCD-E classification, in D3 frequency subband, the minimum coefficient gives the best accuracy of 97.4%. For AB-CD classification, in the D3 frequency subband, approximate entropy gives the maximum accuracy of 82.5%. Moreover, from Table 3, we can infer that the attributes which show the best result for naïve Bayes are Mean Absolute Value and approximate entropy. The maximum accuracy is achieved for A-E and C-E, 100%. The lowest accuracy is achieved for AB-CD classification.

From Table 4, we can observe the results for 16 different classifications for the Decision Tree classifier. For A-E classification, MAV from the D5 frequency subband gives the highest accuracy of 100%. For B-E classification, the maximum coefficient extracted from D3 and D4 and STD extracted from A5 frequency subband give poor results, but MAV extracted from D5 give the best result of 100%. For C-E classification, Shannon entropy extracted from D4 gives the highest accuracy of 98. For D-E classification, in the D3 frequency subband, MAV gives the best accuracy of 96.5%. For AB-E classification, in the D5 frequency subband, MAV gives the maximum accuracy of 100%. For AC-E classification, in the D3 frequency subband, STD provides the highest level of accuracy of 98.67%. In the D5 frequency subband, ApEp provides the highest level of accuracy of 98.67%. For AD-E classification, in the D3 frequency subband, MAV provides the highest accuracy of 98%. For BC-E classification, in the D5 frequency subband, MAV provides the highest level of accuracy of 98.33%. For BD-E classification, in the D5 frequency subband, MAV provides the highest level of accuracy of 94.67%. For CD-E classification, in the D3 frequency subband, MAV provides the highest level of accuracy of 96.67%. For ABC-E classification, in the D3 frequency subband, the minimum coefficient gives the best accuracy of 94.5%. For ABD-E classification, in the D4 frequency subband, the maximum coefficient gives the highest accuracy of 95.75%. For ACD-E classification, in the D3 frequency subband, MAV gives the maximum accuracy of 98%. For BCD-E classification, in the D5 frequency subband, ApEp gives the maximum accuracy of 96.25%. For ABCD-E classification, in the D3 frequency subband, the minimum coefficient gives the best accuracy of 100%. For AB-CD classification, in the D3 frequency subband, MAV gives the maximum accuracy of 79.75%. Moreover, we can infer that the attributes that show the Decision Tree's best result are Mean Absolute Value and Shannon entropy. The highest accuracy is achieved for A-E, B-E, AB-E, and ABCD-E classifications, which is 100%. The lowest classification is performed for AB-CD classification.

### 3.2. Results from Clinical Real-Time Dataset

A real-time clinical dataset from a healthy signal is distinguished from an epileptic patient signal. We have applied DWT and generated the features for different subbands. This work has considered all the 21-channel datasets obtained for 24 sec. The features were generated from subbands D3–D5 and A5, and these features were used for classification [15, 16, 18]. But the better result has been obtained only for the average power feature derived from the D5 subband using the SVM classifier.  Table 5 shows the results. Here, we applied 10-fold cross-validation for classification, since most of the useful information [48] required for distinguishing healthy and seizure patient signals might be in subband D5.

## 4. Comparison with Existing State of the Art

Different researchers had proposed several techniques to detect epileptic seizures from EEG signals. Their works are compared with this work and tabulated in Table 6. The methods that used the same dataset are shown for comparison. It has been noticed that several strategies, such as DTCWT, empirical mode decomposition, CNN, and Fuzzy Neural Network, are used to examine EEG to identify epileptic seizures from normal conditions.

The majority of the researchers classified set A with set E for the two-class classifications and got a classification accuracy from 94.8% to 100% [19–31, 39–42]. Many researchers also classified set B with set E and achieved a classification accuracy from 82.88% to 99.25% [19, 25, 29, 31, 41]. On classifying set C with set E, researchers got a classification accuracy from 88% to 99.6% [23, 25, 29, 31, 41]. For classification of set D with set E, researchers got classification accuracy from 79.94% to 95.85% [23, 25, 29, 31, 41]. We, too, have achieved 100% in A-E classification in our work. We have got better results for B-E, C-E, and D-E classifications. We achieved 100% accuracy for B-E classification, whereas the maximum accuracy to date has been 99.25% only. Similarly, for C-E classification, we achieved 100% accuracy, whereas the maximum accuracy to date has been 99.6% only. We have achieved 97.5% for D-E classification, but the maximum accuracy achieved to date has been 95.85%.

Researchers also combined two datasets from set A to set D and classified them with set E. In the case of AB-E classification, the maximum accuracy achieved to date has been 99.2% [29]. In our work, we have achieved 100% accuracy. Our accuracy is 98.6% for AC-E classification, but the maximum accuracy achieved has been 99.5% [23]. For AD-E classification, researchers got classification accuracy of 85.9% [30] and 97.08% [29], but we got better accuracy of 98%. Researchers got a classification accuracy of 98.25% [31], but we got a better accuracy of 98.67%. In the case of BD-E classification, we got a classification accuracy of 96.33%, but the maximum accuracy achieved has been 96.5% [28]. Similarly, for CD-E classification, we got a classification accuracy of 98%, but the maximum accuracy achieved is 100% [26]. Likewise, researchers have combined three different datasets and classified them with set E. Researchers have achieved a classification accuracy of 98.68% [31] for ABC-E, but we have achieved a better accuracy of 99% in our work. For ACD-E classification, researchers have achieved classification accuracy from 96.65% to 98.15% [20, 25, 31, 34]. We have achieved a slightly better accuracy of 98.25% in our work. We have also classified ABD-E, which has not been computed in any previous work, and have achieved an accuracy of 97%. We have achieved a classification accuracy of 97% for BCD-E classification, but the highest accuracy has been 97.72% [31].

The other two-class classifications are ABCD-E and AB-CD. For ABCD-E classification, our result is comparable with those of other researchers. Researchers have achieved accuracy ranging from 97.1% [28] to 100% [26]. In our work also, we have reached an accuracy of 100%. Additionally, we have combined set A with set B and set C with set D and classified these two combined datasets. This type of classification has not been attempted previously, and we got a classification accuracy of 82.5%.

Furthermore, for three-class classification, AB-CD-E, researchers have achieved classification accuracy ranging from 95.6% to 98.8% [22, 28, 31, 35, 36]. We have got a lesser accuracy of 95% only in our work.

Many studies have been carried out on applying ensemble techniques to various aspects of science and engineering. Ensemble models combine several base models to achieve an overall model with high predictive ability. Ensemble models as used in various areas of science and engineering are provided in [5, 43–45].

### 4.1. Discussion of Key Findings

For A-E classification, MAV, STD, and average power extracted from the D5 frequency subband are fed into kNN, NB, and DT classifiers, giving the best result of 100% accuracy. The SVM classifier gives 100% accuracy for approximate entropy features from the D5 frequency subband. For B-E classification, MAV, STD, and average power taken out from the D5 frequency subband are fed into kNN and DT classifier, which gives the best result of 100% accuracy. For C-E classification, STD and average power extracted from the D3 frequency subband are fed into the NB classifier, giving the best result of 100% accuracy. For D-E classification, MAV extracted from the D3 frequency subband is fed into the NB classifier, which gives the best result of 97.5% accuracy. For AB-E classification, MAV and Shannon entropy extracted from the D5 frequency subband are fed into the kNN and DT classifier, giving the best accuracy result of 100% accuracy. For AC-E classification, STD extracted from the D3 and D5 frequency subbands is fed into kNN and DT classifier, giving the best result of 98.67% accuracy. For AD-E classification, MAV extracted from the D3 frequency subband is fed into all classifiers, giving the best result of 98% accuracy. For BC-E classification, MAV extracted from the D5 frequency subband is fed into kNN, NB, and DT classifier, giving the best result of 98.67% accuracy. For BD-E classification, MAV extracted from the D5 frequency subband is fed into the SVM classifier, giving the best result of 96.33% accuracy. For CD-E classification, MAV extracted from the D3 frequency subband is fed into the SVM classifier, giving the best result of 98% accuracy. For ABC-E classification, MAV extracted from the D5 frequency subband is fed into SVM, kNN, and NB classifier, which gives the best result of 99% accuracy. For ABD-E classification, MAV extracted from the D5 frequency subband is fed into the SVM classifier, which gives the best result of 97% accuracy. For ACD-E classification, MAV extracted from the D3 frequency subband is fed into SVM and NB classifier giving the best result of 98.25% accuracy. For BCD-E classification, MAV extracted from the D5 frequency subband is fed into SVM and NB classifier, which gives the best result of 97% accuracy. For the ABCD-E classification, minimum coefficient extracted from the D5 frequency subband is fed into SVM, kNN, and DT classifier, giving the best result of 100% accuracy. For AB-CD classification, ApEp extracted from the D3 frequency subband is fed into kNN and NB classifier, which gives the best result of 82.5% accuracy. For AB-CD-E classification, Shannon entropy from the D5 frequency subband is fed into the kNN classifier, which gives the best result of 95% accuracy. From Table 6, we can conclude that we have achieved 100% accuracy for A-E, B-E, C-E, AB-E, and ABCD-E classifications, which have been achieved previously. Additionally, we achieved better accuracy for the dataset combinations of D-E, BC-E, and ABC-E in the detection of epileptic seizure.

## 5. Conclusions

A new approach for identifying epileptic seizures by using the time-frequency domain features and various classifiers is proposed in this work. The dataset developed by the University of Bonn in Germany achieves the highest classification rate of 100%. The overall accuracy of 91.67% is obtained in real-time data from the Senthil Multispecialty Hospital, India. The proposed method is successful after verifying and comparing it with the accuracies of the existing methods in several existing literature. The work also presented different base classifier machine learning models to characterize EEG signals and accurately detect epileptic seizures. One of the significant contributions of this work is that if offered wide-ranging machine learning models on the dataset, the proposed method could guarantee accurate prediction. In contrast, other existing works on EEG signals do not examine as many models explored in this work. Examining the different base classifier models is vital for generalization. This is one of the strengths and critical contributions of this paper. Since we could test the validity of the results clinically, we would develop this algorithm further to implement it in the hospitals in our future work.

## Figures and Tables

**Figure 1:** Block diagram of the proposed methodology.

**Figure 2:** Sample EEG signals from datasets A to E.

**Table 1:** SVM results for University of Bonn dataset.

Sets (cases)	Frequency subband	Feature	Classifier accuracy (%)	Sensitivity (%)	Specificity (%)	PPV	NPV	MCC
A-E	D3	Max. coeff.	97	94	100	100	94.84	0.94
	D4	Max. coeff.	98.5	97	100	100	97.2	0.97
	D5	Ap. entropy	100	100	100	100	100	1
	A5	Min. coeff.	94.5	90	99	99.09	91.51	0.89
B-E	D3	Min. coeff.	90	82	98	97.88	85.19	0.81
	D4	Min. coeff.	91	85	97	96.72	87.78	0.83
	D5	Ap. entropy	99.5	99	100	100	99.09	0.99
	A5	Min. coeff.	92	88	96	95.72	89.53	0.81
C-E	D3	MAV	97.5	96	99	99.09	96.36	0.95
	D4	Max. coeff.	98	97	99	99.09	97.42	0.96
	D5	Ap. entropy	98	97	99	99.09	97.42	0.96
	A5	Max. coeff.	79.5	65	94	92.46	74.46	0.62
D-E	D3	MAV	96	94	98	98.18	94.69	0.92
	D4	MAV	94	91	97	97.27	92.07	0.88
	D5	Ap. entropy	93.5	97	90	91.54	97.18	0.87
	A5	Min. coeff.	75.5	66	85	83.87	72.61	0.53
AB-E	D3	Max. coeff.	92	85	95.5	91.18	92.88	0.82
	D4	Min. coeff.	94.66	89	97.5	97.18	94.94	0.88
	D5	Ap. entropy	99.67	100	99.5	99.09	100	0.99
	A5	Min. coeff	95.3	90	98	96.27	95.3	0.89
AC-E	D3	MAV	98.33	96	99.5	99.09	98.13	0.96
	D4	Min. coeff.	94.66	89	97.5	95.2	94.9	0.88
	D5	MAV	98.66	97	99.5	99.09	98.57	0.97
	A5	Min. coeff.	87	83	89	80.02	91.57	0.71
AD-E	D3	MAV	98	96	99	98.18	98.09	0.95
	D4	MAV	96	93	97.5	95.87	96.8	0.91
	D5	MAV	96.66	96	97	94.36	98.1	0.92
	A5	Ap. entropy	84.66	67	93.5	84.68	85.3	0.64
BC-E	D3	Min. coeff.	92.6	86	96	92.02	93.4	0.83
	D4	MAV	93	91	94	98.1	95.6	0.84
	D5	MAV	98.6	97	99.5	99.1	98.54	0.97
	A5	Min. coeff.	86.6	80	90	80	90	0.87
BD-E	D3	Min. coeff.	91.33	86	94	89.5	93.42	0.81
	D4	MAV	92.66	90	94	88.9	95.11	0.84
	D5	MAV	96.3	96	96.5	93.68	97.96	0.92
	A5	Min. Coeff.	82.66	73	87.5	78.17	87.15	0.62
CD-E	D3	MAV	98	97	98.5	97.27	98.61	0.95
	D4	MAV	96.6	93	98.5	97.09	96.6	0.92
	D5	MAV	96.3	95	97	94.42	97.5	0.91
	A5	STD	82.3	61	93	78.75	83.2	0.57
ABC-E	D3	Max. Coeff.	94.5	91	95.6	88.8	97.1	0.86
	D4	MAV	96.6	93	98.5	97.1	96.6	0.92
	D5	MAV	99	97	99.6	99.1	99.1	0.97
	A5	Min. Coeff.	88.5	85	89.6	74.5	95	0.71
ABD-E	D3	Max. Coeff	92.5	87	94.33	84.01	95.6	0.80
	D4	Shannon ent.	95.75	83	100	100	94.74	0.88
	D5	MAV	97	97	97	91.69	99	0.92
	A5	Min. Coeff.	87.75	82	89.66	73.1	93.82	0.69
ACD-E	D3	MAV	98.25	96	99	97.1	98.6	0.95
	D4	STD	97.5	96	98	94.6	98.7	0.93
	D5	MAV	97.25	96	97.66	93.6	98.6	0.93
	A5	STD	86.25	63	94	79.28	88.6	0.61
BCD-E	D3	Min. Coeff.	92.75	83	96	94.60	89.55	0.81
	D4	Shannon ent.	94.5	80	99.33	93.87	97.87	0.85
	D5	MAV	97	96	97.33	98.66	98.6	0.92
	A5	STD	85.75	63	93.33	88.43	88.43	0.60
ABCD-E	D3	Min. Coeff.	100	100	100	100	100	1
	D4	Shannon ent.	87.4	51	96.5	79.9	88.9	0.56
	D5	MAV	97.4	97	97.5	90.87	99.25	0.922
	A5	Shannon ent.	88.2	57	96	79.2	90.00	0.60
AB-CD	D3	Approx. Ent.	80	76.5	83.5	83.09	78.5	0.60
	D4	Approx. Ent.	64.5	42	87	78.6	60.2	0.33
	D5	Min. Coeff.	72.5	71	74	73.9	72.02	0.45
	A5	Approx. Ent.	69.75	68	71.5	70.7	69.6	0.391

Ap. entropy: approximate entropy; Max. coeff.: maximum coefficient; MAV: mean absolute value; Approx. entropy: approximate entropy.

**Table 2:** kNN results for University of Bonn dataset.

Sets (cases)	Frequency subband	Feature	Classifier accuracy (%)	Sensitivity (%)	Specificity (%)	PPV	NPV	MCC
A-E	D3	Max. coeff.	97	94	100	100	94.84	0.94
	D4	Min. coeff.	98.5	97	100	100	97.27	0.97
	D5	Ap. entropy	100	100	100	100	100	1
	A5	Min. coeff.	94.5	90	99	99.09	91.51	0.89
B-E	D3	Max. coeff.	92.5	90	95	95.55	91.36	0.85
	D4	Min. coeff.	93.5	91	96	96.07	92.56	0.87
	D5	MAV	100	100	100	100	100	1
	A5	Min. coeff.	93.5	91	96	96.09	92.11	0.87
C-E	D3	STD	98	98	98	98.18	98.1	0.96
	D4	STD	98	98	98	98.1	98.1	0.96
	D5	MAV	98	97	99	99.1	97.3	0.96
	A5	Approx. ent	79.5	75	84	82.8	77.6	0.59
D-E	D3	MAV	97	97	97	97.1	97.1	0.94
	D4	Shannon ent.	95	96	94	94.4	96.1	0.90
	D5	MAV	93.5	94	93	93.8	94.5	0.87
	A5	Max. coeff.	73	72	74	75.2	73.5	0.47
AB-E	D3	Max. coeff.	95.6	88	99.5	98.8	94.4	0.9
	D4	Max. coeff.	93.6	92	94.5	90.8	96	0.86
	D5	MAV	100	100	100	100	100	1
	A5	Min. coeff.	93.6	87	97	94.3	94.1	0.86
AC-E	D3	STD	98.7	98	99	98.1	99.1	0.97
	D4	Max. coeff.	93.7	92	94.5	91	95.9	0.86
	D5	MAV	98.7	97	99.5	99.1	98.6	0.97
	A5	Ap. entropy	85	71	93	86.3	87.02	0.68
AD-E	D3	MAV	98	97	98.5	97.18	98.54	0.95
	D4	MAV	95.3	93	96.5	93.73	96.61	0.89
	D5	MAV	95.7	94	96.5	93.59	97.03	0.90
	A5	Min. coeff.	80.7	67	87.5	73.42	84.39	0.56
BC-E	D3	Max. coeff.	95.33	88	99	98.09	94.59	0.89
	D4	MAV	94	88	97	93.95	94.32	0.84
	D5	MAV	98.66	97	99.5	99.09	98.61	0.97
	A5	Ap. entropy	85.33	73	91.5	82.47	87.72	0.67
BD-E	D3	Max. coeff.	93.33	88	96	92.32	94.22	0.85
	D4	MAV	94.66	88	98	95.72	94.41	0.88
	D5	Shannon ent.	95.33	95	95.5	91.43	97.57	0.89
	A5	Min. coeff.	81	70	86.5	74.02	85.32	0.57
CD-E	D3	MAV	97.66	96	98.5	97.33	98.07	0.94
	D4	MAV	94.66	92	96	92.78	92.78	0.88
	D5	MAV	95.33	94	96	92.54	92.54	0.89
	A5	Ap. entropy	80	65	87.5	74.03	83.33	0.54
ABC-E	D3	Max. coeff.	94.5	89	98.33	95.78	96.57	0.89
	D4	MAV	94.66	92	96	92.78	96.15	0.88
	D5	MAV	99	97	99.66	99.09	99.05	0.97
	A5	Min. coeff	88.25	70	94.33	80.65	90.53	0.67
ABD-E	D3	Min. coeff.	91.75	80	95.66	87.18	93.56	0.78
	D4	MAV	95.75	88	98.33	95.78	96.25	0.88
	D5	MAV	96.5	94	97.33	92.29	98.06	0.90
	A5	Ap. entropy	86.25	68	92.33	77.01	89.89	0.63
ACD-E	D3	Shannon ent.	98	97	98.33	95.27	98.98	0.94
	D4	Shannon ent.	97.25	96	97.66	94.20	98.7	0.93
	D5	STD	96.25	93	97.33	92.82	97.73	0.90
	A5	Ap. entropy	85.5	65	92.33	74.76	88.97	0.60
BCD-E	D3	Max. coeff.	93.5	84	96.66	89.63	94.83	0.82
	D4	STD	94.25	85	97.33	92.16	95.15	0.84
	D5	MAV	96.5	94	97.33	92.87	98.08	0.91
	A5	Ap. entropy	85.5	64	92.66	76.47	88.62	0.60
ABCD-E	D3	Min. Coeff.	100	100	100	100	100	1
	D4	Avg power	88.4	60	95.5	76.85	90.74	0.60
	D5	MAV	97	93	98	92.72	98.3	0.90
	A5	Avg power	88	59	95.25	75.84	90.39	0.59
AB-CD	D3	Ap. entropy	82.5	70	95	93.09	76.56	0.67
	D4	MAV	59.75	56.5	63	60.9	59.09	0.19
	D5	MAV	75	59.5	90.5	86.52	69.21	0.52
	A5	Ap. entropy	73.25	51	95.5	92.79	66.59	0.52
AB-CD-E	D3	MAV	73.8	74	73.75	42.47	91.87	0.40
	D4	MAV	64.2	85	59	34.21	94.17	0.35
	D5	Shannon ent.	75	95	70	44.82	98.35	0.52
	A5	Ap. entropy	66.4	65	66.75	33.23	88.37	0.26

Ap. entropy: approximate entropy; Min. coeff.: minimum coefficient, MAV: mean absolute value; Approx. entropy: approximate entropy; Shannon ent.: Shannon entropy; STD: standard deviation.

**Table 3:** Naïve Bayes results for University of Bonn dataset.

Sets (cases)	Frequency subband	Feature	Classifier accuracy (%)	Sensitivity (%)	Specificity (%)	PPV	NPV	MCC
A-E	D3	STD	99.5	99	100	100	99.09	0.99
	D4	MAV	99.5	99	100	100	99.09	0.99
	D5	MAV	100	100	100	100	100	1
	A5	Min. coeff.	93.5	91	96	96.33	92.35	0.87
B-E	D3	Min. coeff.	90.5	83	98	98	86.07	0.82
	D4	Avg. power	92.5	86	99	98.88	89.05	0.86
	D5	MAV	99.5	100	99	99.09	100	0.99
	A5	Ap. entropy	92	87	97	97.09	89.08	0.85
C-E	D3	STD	100	100	100	100	100	1
	D4	STD	98	98	98	98.18	98.18	0.96
	D5	STD	98	97	99	99.09	99.09	0.96
	A5	STD	79.5	62	97	94.90	72.96	0.63
D-E	D3	MAV	97.5	97	98	98.18	97.27	0.95
	D4	MAV	94	91	97	97.18	92.98	0.88
	D5	Ap. entropy	94	97	91	92.03	97.18	0.88
	A5	Min. coeff.	75	60	90	88.86	70.34	0.54
AB-E	D3	Min. coeff.	93	85	97	94.62	93.08	0.84
	D4	MAV	94.33	90	96.5	93.58	95.22	0.87
	D5	STD	99.7	100	99.5	99.09	100	0.99
	A5	Min. coeff.	94	86	98	96.22	93.52	0.86
AC-E	D3	STD	98.7	98	99	98.18	99.04	0.97
	D4	MAV	94.3	90	96.5	93.58	95.22	0.87
	D5	Ap. ent.	98.7	98	99	98.1	99.02	0.97
	A5	STD	86.7	65	97.5	93.35	84.88	0.69
AD-E	D3	MAV	98	96	99	98.33	98.09	0.95
	D4	MAV	96.3	93	98	96.27	96.71	0.92
	D5	Ap. ent.	95.7	97	95	91.54	98.54	0.91
	A5	Min. coeff.	82.7	60	94	84.38	82.86	0.59
BC-E	D3	Min. coeff.	93.3	83	98.5	97.07	92.3	0.85
	D4	MAV	94.7	90	97	93.91	95.4	0.88
	D5	Ap. ent.	98.7	97	99.5	99.10	98.5	0.97
	A5	Max. coeff.	80.3	64	97.5	93.25	84.7	0.68
BD-E	D3	Max. coeff.	90	74	98	95.5	88.56	0.77
	D4	MAV	93.3	85	97.5	94.75	93.04	0.85
	D5	Ap. ent.	96	97	95.5	92.43	98.43	0.91
	A5	Min. coeff.	83.3	60	95	86.46	83.17	0.61
CD-E	D3	MAV	97.7	97	98	96.27	98.54	0.94
	D4	MAV	97.7	93	98.5	96.72	96.73	0.92
	D5	Ap. ent.	96	97	95.5	92.09	98.52	0.91
	A5	Min. coeff.	82.3	55	96	65.82	81.88	0.59
ABC-E	D3	Min. coeff.	94.5	85	97.67	94.02	95.33	0.85
	D4	MAV	96.67	93	98.5	96.72	96.73	0.92
	D5	MAV	99	98	99.33	98.18	99.35	0.97
	A5	Max. coeff.	89.75	64	98.33	93.67	89.47	0.70
ABD-E	D3	Min. coeff.	93.25	79	98	93.41	93.42	0.81
	D4	Avg power	95.75	92	97	92.52	97.39	0.89
	D5	Ap. ent.	96.25	93	97.3	92.66	97.71	0.90
	A5	Min. Coeff.	87.25	60	96.3	84.76	88.05	0.63
ACD-E	D3	MAV	98.25	96	99	97.27	98.72	0.95
	D4	STD	97.25	94	98.3	95.42	98.10	0.92
	D5	Ap. ent.	97	97	97	91.87	98.97	0.92
	A5	Min. coeff.	87.25	57	97.3	86.88	87.48	0.63
BCD-E	D3	Min. coeff.	93	78	98	92.67	93.23	0.80
	D4	MAV	95	88	97.3	91.84	96.11	0.86
	D5	Ap. ent.	97	97	97	91.87	98.99	0.92
	A5	Min. coeff.	87.25	89	96.67	87.87	87.75	0.90
ABCD-E	D3	Min. coeff.	97.4	87	100	100	96.89	0.91
	D4	Min. coeff.	89.8	60	97.25	85.51	90.81	0.65
	D5	Ap. ent.	97.6	97	97.25	91.8	99.24	0.92
	A5	Min. coeff.	90	60	97.5	86.09	90.78	0.66
AB-CD	D3	Ap. ent.	82.5	70	95	93.09	76.56	0.67
	D4	Ap. ent.	64.5	42	87	78.68	60.23	0.33
	D5	MAV	74	53.5	94.5	90.62	67.32	0.52
	A5	MAV	74	53.5	94.5	90.62	67.32	0.52

Ap. entropy: approximate entropy; MAV: mean absolute value; STD: standard deviation.

**Table 4:** Decision Tree results for University of Bonn dataset.

Sets (cases)	Frequency subband	Feature	Classifier accuracy (%)	Sensitivity (%)	Specificity (%)	PPV	NPV	MCC
**A-E**	D3	Avg. power	99	99	100	100	99.09	0.99
	D4	MAV	99.5	99	100	99.09	99.09	0.99
	**D5**	**MAV**	**100**	**100**	**100**	**100**	**100**	**1**
	A5	Min. coeff.	92.5	92	93	93.54	92.38	0.85
B-E	D3	Max. coeff.	91.5	88	95	95.45	91.21	0.84
	D4	Max. coeff.	90.5	89	92	92.4	89.8	0.81
	**D5**	**MAV**	**100**	**100**	**100**	**100**	**100**	**1**
	A5	STD	89.5	91	88	89.23	92.17	0.8
C-E	**D3**	**STD**	**98**	**98**	**98**	**98.18**	**98.18**	**0.96**
	**D4**	**Shannon ent.**	**98**	**98**	**98**	**98.33**	**98.18**	**0.96**
	D5	MAV	97.5	97	98	99.09	97.27	0.96
	A5	Max. coeff.	80	77	83	82.47	79.25	0.6
D-E	D3	MAV	96.5	97	96	96.27	97.18	0.93
	D4	MAV	92.5	93	92	92.87	93.16	0.85
	D5	MAV	91.5	91	92	93.09	91.91	0.83
	A5	Max. coeff.	69	70	68	69.35	69.8	0.38
AB-E	D3	Max. coeff.	92.67	88	95	91.09	94.35	0.84
	D4	MAV	94.33	87	98	96.5	94.11	0.87
	**D5**	**MAV**	**100**	**100**	**100**	**100**	**100**	**1**
	A5	Min. coeff.	92	87	94.5	89.28	93.83	0.82
AC-E	**D3**	**STD**	**98.67**	**98**	**99**	**98.18**	**99.04**	**0.97**
	D4	MAV	94.33	90	96.5	93.58	95.22	0.87
	**D5**	**Ap. ent.**	**98.67**	**98**	**99**	**98.1**	**99.02**	**0.97**
	A5	STD	86.67	89	97.5	93.35	84.88	0.69
AD-E	**D3**	**MAV**	**98**	**97**	**98.5**	**97.18**	**98.54**	**0.95**
	D4	MAV	94.3	92	95.5	91.47	96.15	0.87
	D5	Ap. ent.	94.67	91	96.5	93	95.7	0.88
	A5	Min. coeff.	81.33	72	86	73.64	86.81	0.59
BC-E	D3	Max. coeff.	93.67	87	97	95.1	93.85	0.86
	D4	MAV	93.3	88	96	93.28	94.39	0.85
	**D5**	**MAV**	**98.33**	**97**	**99**	**98.18**	**98.57**	**0.96**
	A5	Ap. ent.	81.67	71	87	76.02	85.68	0.59
BD-E	D3	Max. coeff.	88.3	82	91.5	84.34	91.31	0.74
	D4	MAV	91.67	88	93.5	87.94	94.08	0.81
	**D5**	**MAV**	**94.67**	**92**	**96**	**93.09**	**96.33**	**0.88**
	A5	Min. coeff.	80.33	70	85.5	73.41	85.46	0.56
CD-E	**D3**	**MAV**	**96.67**	**97**	**96.5**	**94.11**	**98.54**	**0.93**
	D4	MAV	94	93	94.5	90.18	96.64	0.87
	D5	Ap. ent.	94	92	95	90.75	96.37	0.86
	A5	Min. coeff.	76.66	65	82.5	65.82	82.73	0.47
ABC-E	**D3**	**Min. coeff**.	**94.5**	**87**	**97**	**90.86**	**95.97**	**0.85**
	D4	MAV	94	93	94.5	90.18	96.65	0.87
	D5	MAV	98.5	96	99.3	98.18	98.72	0.96
	A5	Max. coeff.	89.75	68	99.1	87.32	90.43	0.7
ABD-E	D3	Min. coeff.	92.5	84	95.33	86.32	94.76	0.8
	**D4**	**Max. coeff.**	**95.75**	**90**	**97.66**	**93.61**	**96.75**	**0.8**
	D5	Ap. ent.	95.25	90	97	91.68	96.85	0.87
	A5	Min. coeff.	85.75	72	90.3	72.18	90.86	0.62
ACD-E	**D3**	**MAV**	**98**	**97**	**98.33**	**95.75**	**99.05**	**0.95**
	D4	STD	96.75	96	97	91.81	98.6	0.91
	D5	Ap. ent.	95.5	91	97	92.18	97.13	0.88
	A5	MAV	82.25	66	87.66	63.85	88.75	0.53
BCD-E	D3	Min. coeff.	91.25	85	93.33	81.72	94.93	0.77
	D4	Avg. power	94.25	85	97.33	91.77	95.17	0.84
	**D5**	**Ap. ent.**	**96.25**	**95**	**96.6**	**91.2**	**98.35**	**0.9**
	A5	STD	82.75	63	89.33	68	88.15	0.53
ABCD-E	D3	Min. coeff.	100	100	100	100	100	1
	D4	Min. coeff.	85.8	65	91	64.72	91.29	0.55
	D5	Ap. ent.	96.8	95	97.25	90.93	98.75	0.9
	A5	Avg. power	85.2	58	92	63.43	89.86	0.51
AB-CD	**D3**	**MAV**	**79.75**	**74.5**	**85**	**84.23**	**77.09**	**0.63**
	D4	Avg. power	57.75	56.5	59	58.15	57.95	0.15
	D5	Min. coeff.	73.5	68	79	76.59	72.88	0.48
	A5	Avg. power	74	52	96	93.62	67.06	0.53

**Table 5:** Results for real-time clinical datasets using average power feature for different classifiers.

Sets (cases)	Classifier	Classifier accuracy (%)	Sensitivity (%)	Specificity (%)	PPV	NPV	MCC
Healthy versus epileptic patients	SVM	91.667	83.33	100	100	87.5	0.85
	kNN	75	50	100	100	67.5	0.58
	Naïve Bayes	75	100	50	75	0	0
	Decision Tree	50	0	100	0	50	0

SVM: support vector machine.

**Table 6:** Comparison with the existing state of the art.

References	Year	Methods	Cases	CA (%)
[30]	2006	DWT adaptive neurofuzzy network	AD-E	85.9
[31]	2009	DWT + ApEn and surrogate data analysis	ACD-E	96.65
[18]	2010	Line length feature and ANN	A-E	99.6
			ACD-E	97.75
			ABCD-E	97.5
[20]	2011	Statistical features from DWT + kNN classifier	A-E	100.0
			AB-CD-E	95.6
[21]	2012	Permutation entropy + SVM	A-E	100.0
			B-E	82.88
			C-E	88.0
			D-E	79.94
[32]	2012	Statistical features from DWT + PCA + ANN classifier	A-E	100.0
[17]	2012	ApEp + SampEp + phase entropy 1 + phase entropy 2-Fuzzy Sugeno classifier	AB-CD-E	98.1
[29]	2013	DWT + permutation and sample entropy + Hurst exponent + genetic algorithm + extreme learning machine (ELM)	A-E	94.8
[34]	2013	DWT + Hurst and Lyapunov exponent	B-E	96.5
[24]	2014	Dual-tree complex wavelet transform + kNN transform	A-E	100.0
			CD-E	100.0
			ABCD-E	100.0
[25]	2015	Empirical mode decomposition-based temporal spectral features + SVM	A-E	100.0
[26]	2015	DTCWT + complex-valued neural network	AB-CD-E	98.28
[33]	2016	DTCWT + general regression neural network	A-E	100.0
			B-E	98.9
			C-E	98.7
			D-E	93.3
			AB-E	99.2
[28]	2016	Key-point based local binary pattern of EEG signals	CD-E	99.45
			AB-CD-E	98.8
[35]	2017	Tunable-Q wavelet transform + kNN entropy + SVM	AB-CD-E	98.6
[4]	2016	DWT – MVP + SD + AVP – NB/kNN classifier	A-E	100.0
			B-E	99.25
			C-E	99.5
			D-E	95.62
			AB-E	99.16
			AC-E	99.5
			AD-E	97.08
			BC-E	98.25
			BD-E	96.5
			CD-E	98.75
			ABC-E	98.68
			ACD-E	97.31
			BCD-E	97.72
			ABCD-E	97.1
[36]	2018	CNN	AB-CD-E	88.67
[37]	2018	CNN	A-E	100
			B-E	99.8
			C-E	99.1
			D-E	99.4
			AB-E	99.8
			AC-E	99.7
			BC-E	99.5
			BD-E	99.6
			CD-E	99.7
			ABC-E	99.97
			ACD-E	99.8
			BCD-E	99.3
			ABCD-E	99.7
			AB-CD	99.9
			AB-CD-E	99.1
			AB-CDE	99.7
This work (University of Bonn dataset)	2020	DWT + SVM/KNN/NB/DT	A-E	**100.0**
			B-E	**100.0**
			C-E	**100.0**
			D-E	97.5
			AB-E	100.0
			AC-E	98.67
			AD-E	98.0
			BC-E	98.67
			BD-E	96.33
			CD-E	98.0
			ABC-E	99.0
			ABD-E	97.0
			ACD-E	98.25
			BCD-E	97.0
			ABCD-E	**100.0**
			AB-CD	82.5
			AB-CD-E	95.0
This work (real-time clinical dataset)	2020	DWT + SVM/KNN/NB/DT	Healthy- epileptic patient	**91.67**

## Data Availability

The data that support the findings of this study are available from the corresponding author upon reasonable request.
